The article "Comprehensive Analysis of Immunoinhibitors Identifies LGALS9 and TGFBR1 as Potential Prognostic Biomarkers for Pancreatic Cancer" was published in 2020. Journal: Comput Math Methods Med.

# Comprehensive Analysis of Immunoinhibitors Identifies LGALS9 and TGFBR1 as Potential Prognostic Biomarkers for Pancreatic Cancer

**DOI:** 10.1155/2020/6138039

**Published:** 2020-09-30

**Authors:** Yue Fan, Tianyu Li, Lili Xu, Tiantao Kuang

**Affiliations:** ^1^Department of Integrated TCM & Western Medicine, Zhongshan Hospital, Fudan University, Shanghai 200032, China; ^2^Department of General Surgery, Zhongshan Hospital, Fudan University, Shanghai 200032, China

## Abstract

Pancreatic cancer (PC) is one of the most deadly cancers worldwide. To uncover the unknown novel biomarker used to indicate early diagnosis and prognosis in the molecular therapeutic field of PC is extremely of importance. Accumulative evidences indicated that aberrant expression or activation of immunoinhibitors is a common phenomenon in malignances, and significant associations have been noted between immunoinhibitors and tumorigenesis or progression in a wide range of cancers. However, the expression patterns and exact roles of immunoinhibitors contributing to tumorigenesis and progression of pancreatic cancer (PC) have not yet been elucidated clearly. In this study, we investigated the distinct expression and prognostic value of immunoinhibitors in patients with PC by analyzing a series of databases, including TISIDB, GEPIA, cBioPortal, and Kaplan-Meier plotter database. The mRNA expression levels of IDO1, CSF1R, VTCN1, KDR, LGALS9, TGFBR1, TGFB1, IL10RB, and PVRL2 were found to be significantly upregulated in patients with PC. Aberrant expression of TGFBR1, VTCN1, and LGALS9 was found to be associated with the worse outcomes of patients with PC. Bioinformatics analysis demonstrated that LGALS9 was involved in regulating the type I interferon signaling pathway, interferon-gamma-mediated signaling pathway, RIG-I-like receptor signaling pathway, NF-kappa B signaling pathway, cytosolic DNA-sensing pathway, and TNF signaling pathway. And TGFB1 was related to mesoderm formation, cell matrix adhesion, TGF-beta signaling pathway, and Hippo signaling pathway. These results suggested that LGALS9 and TGFBR1 might serve as potential prognostic biomarkers and targets for PC.

## 1. Introduction

The mortality of pancreatic cancer (PC), the fourth widely occurred cancer with poor prognosis, has an overall five-year survival rate lower than 10% [1]. Due to the hidden symptoms at early stages, fewer than 15% of patients are diagnosed with PC at a stage when they could be eligible for curative surgical resection [2]. To improve early detection and prognosis and to provide timely and effective treatment for high-risk patients, predictive biomarkers for PC are required [3, 4]. To date, carbohydrate antigen 199 (CA199) and CA242, which are currently used in clinical settings as serum biomarkers for PC, are inadequate for early screening and prognosis [5, 6]. To uncover the unknown novel biomarker used to indicate early diagnosis and prognosis in the molecular therapeutic field of PC is extremely of importance.

Previously, the application of the immune system to recognize and eradicate tumors has made significant advance in the clinical use of cancer immunotherapy [7–9]. Notably, the emergence of immune checkpoints inhibitors typically interfered negative regulators of T cell immunity including LAG3 [10–12], CTLA-4 [13, 14], PD-1 [15, 16], and TIM3 [17, 18]. The advent of these “checkpoint inhibitors” has thoroughly altered and improved the former therapies for melanoma, lung cancer, and so on [19]. For instance, interference of LAG3 relieved the exhaustion of T cells and heightened immunity against tumor due to the interaction among LAG3 with MHC class II and galectin 3 [20]. Additionally, tumor-infiltrating lymphocyte- (TIL-) produced TIM3 has been identified to display a key role in maintaining inactive lymphocyte status or inducing lymphocyte apoptosis [21]. LGALS9 is a ligand of TIM-3 and expressed in a variety of cell types, especially in lymphoid organs and monocytes [22]. In addition, LGALS9 could impose unequal effects on immune cells in a tumor microenvironment [22]. TGF-*β* signaling exhibited importance in biological signal regulation including cell growth and death, differentiation, angiogenesis, and inflammation [23]. Several recent studies demonstrated that TGF-*β* signaling played a key role in immune response [24]. Understanding the potential functions and expression pattern of immune “checkpoint inhibitors” could be helpful for the identification of novel prognosis and treatment biomarkers for PC.

The occurrence and progression of newly produced strategies, comprising microarray and RNA-sequencing, exerted a positive effect in molecular research and also gave impetus to exploring accurate and safe treatment for PC [25–27]. Here, we expanded PC-related knowledge in view of different databases, thus generating a conclusive analysis of the link between the function of immune checkpoint inhibitors and the diagnosis along with the development of PC.

## 2. Materials and Methods

### 2.1. Survival Analysis

Kaplan-Meier plotter (http://www.kmplot.com/) is an online database containing microarray gene expression data, and survival information derived from Gene Expression Omnibus, TCGA, and the Cancer Biomedical informatics Grid. Kaplan-Meier (K-M) Plotter database was used to analyze prognostic parameter of expected candidates [28]. K-M survival curves and logrank test were performed to disintegrate correlation, such as gene expression with overall survival (OS) or first progression (FP) or post progression survival (PPS), respectively. Significant difference was indicated as *P* < 0.05.

### 2.2. Construction of Protein Interaction Network

A functional protein interaction network was constructed as indicated in website (http://string-db.org/) [29]. Among them, 50 selected proteins indeed associating with Homo sapiens were selected, followed by calculating confidence score as more than 0.9.

### 2.3. TISIDB, GEPIA, TCGA, and CBioPortal Analysis

TISIDB is an integrated repository portal for tumor-immune system interactions. The present study used TISIDB (http://cis.hku.hk/TISIDB) database to detect the relationship between centromere protein expression and clinical stages, lymphocytes, immunomodulators, and chemokines in PC. Gene Expression Profiling Interactive Analysis (GEPIA) [30] was a powerful tool to determine key interactive and customizable functions including differential expression analysis, profiling plotting, correlation analysis, patient survival analysis, similar gene detection, and dimensionality reduction analysis, which was used to determine mRNA expression in 9,736 tumors and 8,587 normal tissues. The cBioPortal system was used to investigate cancer genomic and clinical-related characters within 105 cancer subjects in the TCGA pipeline cancer [31]. Besides, the coexpression and interaction of selected proteins were probed referred to cBioPortal guidelines [32].

### 2.4. Gene Ontology and Pathway Enrichment Analysis

Gene ontology (GO) and Kyoto Encyclopedia of Genes and Genomes (KEGG) pathway enrichment analysis was performed using DAVID online tool. *P* < 0.01 was set as the cutoff criterion.

### 2.5. Statistical Analysis

Student's *t*-test was analyzed for statistical significance. Statistical analysis was performed by SPSS 21.0 (SPSS Inc., Chicago, IL).

## 3. Results

### 3.1. Identification of Immunoinhibitor Expression Pattern in PC

The present study analyzed the expression pattern of 23 immunoinhibitors in PC using TCGA database, including CD160, CD244, KIR2DL1, KIR2DL3, BTLA, CSF1R, HAVCR2, TIGIT, LAG3, PDCD1, VTCN1, PDCD1LG2, LGALS9, CD96, TGFBR1, TGFB1, CTLA4, ADORA2A, PVRL2, IL10, IDO1, IL10RB, and KDR. As shown in Figure 1, we found that IDO1, CSF1R, VTCN1, KDR, LGALS9, TGFBR1, TGFB1, IL10RB, and PVRL2 were highly expressed in PC tissues.

### 3.2. Increasing Expression of Immunoinhibitors Was Observed in PC Samples

The GEPIA database was used to compare the difference of expression of 9 overexpressed immunoinhibitors in transcription level between cancers and normal tissues (Figure 1). The data demonstrated TGFB1 (Figure 2(a)), PVRL2 (Figure 2(b)), CSF1R (Figure 2(c)), TGFBR1 (Figure 2(d)), VTCN1 (Figure 2(e)), LGALS9 (Figure 2(f)), IL10RB (Figure 2(g)), KDR (Figure 2(h)), and IDO1 (Figure 2(i)) mRNA levels were significantly upregulated in patients with PC compared to normal tissues.

### 3.3. Immunoinhibitors Were Positively Correlated to the Advanced Stage and Grade in PC

Furthermore, the TISIDB database analysis showed TGFB1 was positively correlated to the advanced grades of PC samples (Figure 3). However, we did not observe a significant upregulation of PVRL2 (Figure 3(b)), CSF1R (Figure 3(c)), TGFBR1 (Figure 3(d)), VTCN1 (Figure 3(e)), LGALS9 (Figure 3(f)), IL10RB (Figure 3(g)), KDR (Figure 3(h)), and IDO1 (Figure 3(i)) in advanced grades of PC samples.

Interestingly, our data also revealed the correlation between Immunoinhibitors level and stages of PC samples. The results displayed that expression of VTCN1 was raised in grade 2 and grade 3 samples compared to grade 1 PC samples, but expression of VTCN1 was decreased in grade 4 sample after being normalized to that in grade 1/2 PC samples (Figure 4(b)). Meanwhile, our data showed IL10RB was enhanced in grade 2, grade 3, and grade 4 PC samples compared to grade 1 PC samples (Figure 4(g)). However, no obvious difference between the expression of TGFB1 (Figure 4(a)), PVRL2 (Figure 4(b)), CSF1R (Figure 4(c)), TGFBR1 (Figure 4(d)), LGALS9 (Figure 4(f)), KDR (Figure 4(h)), and IDO1 (Figure 4(i)) and the stage in the PC patients was taken on.

### 3.4. Analysis of Immunoinhibitor Feature in Prognostic PC Patients

We deeply explored the profile of immunoinhibitors implicated in prognostic PC patients. Our data revealed that the increasing level of TGFBR1 (Figure 5(d)), VTCN1 (Figure 5(e)), LGALS9 (Figure 5(f)), and IDO1 (Figure 5(i)) mRNA was closely pertained to poor OS. However, the dysregulation of TGFB1 (Figure 5(a)), PVRL2 (Figure 5(b)), CSF1R (Figure 5(c)), IL10RB (Figure 5(g)), and KDR (Figure 5(h)) was not related with OS in PC.

### 3.5. To Assess the Coexpression and Interaction Gene with Immunoinhibitors in PC Patients

We evaluated the association of candidate gene expression with immunoinhibitors by Pearson's correlation analysis. The immunoinhibitor-target pair with absolute Pearson's correlation coefficient value > 0.5 was considered significant. The networks were constructed using Cytoscape software. As presented in Figure 6, the coexpression network included 9 immunoinhibitors, 1250 targets, and 1304 edges. From the analysis, we observed LGALS9 may have a primary role in this network and possessed approximately 30% coexpressing targets with IL10RB, PVRL2, and IDO1.

### 3.6. Assessment of the Function of LGALS9 and TGFB1 in PC Patients

We finally validated the role of LGALS9 and TGFB1 after the analysis of GO and KEGG in the DAVID system using their genes. After bioinformatics analyzing, LGALS9 was involved in regulating type I interferon signaling pathway, defense response to virus, interferon-gamma-mediated signaling pathway, response to virus, innate immune response, and negative regulation of viral genome replication (Figure 7(a)). KEGG pathway analysis demonstrated that LGALS9 was related to the RIG-I-like receptor signaling pathway, NF-kappa B signaling pathway, cytosolic DNA-sensing pathway, and TNF signaling pathway (Figure 7(b)).

Also, we found that TGFB1 was related to mesoderm formation, cell matrix adhesion, substrate adhesion-dependent cell spreading, in utero embryonic development, extracellular matrix organization, outflow tract septum morphogenesis, mitral valve morphogenesis, and Hippo signaling (Figure 7(c)). And KEGG pathway analysis showed TGFB1 was related to pathways in cancer, TGF-beta signaling pathway, focal adhesion, signaling pathways regulating pluripotency of stem cells, regulation of actin cytoskeleton, Hippo signaling pathway, and shigellosis (Figure 7(d)).

## 4. Discussion

PC with a poor prognosis was regarded as one of the most deadly carcinomas [33]. The growth and development of Cancer were reported to be involved in the process of immune suppression [34]. Cancer cells could stimulate various immune checkpoint pathways responsible for curbing immunity [35]. Monoclonal antibodies targeting immune checkpoints exhibited huge advance in cancer therapy. Currently, some researches have revealed that patients with different cancer recovered better after treatment of immunoinhibitors. Developing prospective methods based on immunoinhibitors could be of significance to explore novel biomarkers in the PC diagnosis and prognosis.

In this study, we analyzed the expression pattern of 23 immunoinhibitors in PC using TCGA database and found that IDO1, CSF1R, VTCN1, KDR, LGALS9, TGFBR1, TGFB1, IL10RB, and PVRL2 were highly expressed in PC tissues. Moreover, the analysis revealed that IDO1, CSF1R, VTCN1, KDR, LGALS9, TGFBR1, TGFB1, IL10RB, and PVRL2 mRNA level was significantly upregulated in patients with PC compared to normal tissues. Kaplan-Meier plotter results demonstrated that the increasing level of TGFBR1, VTCN1, and LGALS9 mRNA was closely pertained to poor OS.

TGF-*β* was a primary executor of the stability and tolerance of the internal environment of immune system, including controlling many component functions [36]. Thus, disrupting TGF-*β* signal could result in inflammatory diseases and tumorigenesis. In addition, TGF-*β* is also a preliminary immunosuppressor in the tumor microenvironment [37]. Current researches have reported TGF-*β* was engaged in tumor immune evasion and adverse reactions to tumor immunotherapy [37]. Nevertheless, our study confirmed that TGFBR1 and TGFB1 are upregulated in PC samples. Kaplan-Meier analysis showed that TGFBR1 was associated with reduced OS and PFS time in PC patients.

VTCN1 exists on the surface of antigen-presenting cells (APC) and interacts with ligands that bind to T-cell surface receptors [38]. The activity of B7-H4 was illustrated to be related to the reduced inflammatory CD4^+^ T cell response as previously described. Studies have indicated VTCN1 expression was positively linked to tumor progression and acted as a candidate for the treatment of cancer [39]. The level of B7-H4 on tumor cells with adverse clinical and pathologic features endowed B7-H4 with clinical significance [40]. Moreover, the expression of B7-H4 in tumor-associated macrophages was correlated with Foxp3^+^ regulatory T cells (Tregs) [41]. Because the expression of B7-H4 was on a variety of tumor cells and tumor-related macrophages, blocking of B7-H4 could improve the tumor microenvironment, thus enabling antigen-specific clearance of tumor cells [41]. Our study suggested the enhanced level of VTCN1 was related to OS time and PFS (progression-free survival) time of PC. Nevertheless, no increasing level of VTCN1 was shown in neither PC nor normal tissues.

Transmembrane receptor TIM-3 was encoded by *HAVCR2* and expressed on a variety of cells [42]. The expression of TIM-3 is closely related to exhaustion and impaired function of T cells. The interaction between TIM-3 and galectin 9 has been demonstrated to induce Th1 cell apoptosis, leading to reduced responses from autoimmunity and antitumor immunity [22] and also making TIM-3 as a potential target for ICB. Of note, our study firstly exposed the upregulated level of LGALS9 in PC patients was associated with shorter OS and PFS time.

IDO1 was responsible for converting tryptophan (Trp) into downstream catabolic product, called caninuria. Emerging studies have shown that IDO1 was expressed in a large number of human cancers. In the transcription level, IDO1 displayed powerful relevance with T cell infiltration [43].

Even though the expression of CSFR1, KDR, IL10RB, and PVRL2 was upregulated in PC samples, which was not associated with the prognosis of PC. CSFR1 was mostly found in aggressive cell models and participated in the invasion and migration of tumor cells, and its expression is related to the poor prognosis of cancer patients. Positive feedback existed between the expressions of CSF1 and EGF in tumors [44]. By blocking the signal transduction mediated by the EGF receptor or CSF-1 receptor, incomplete feedback loop would inhibit the migration and invasion of macrophages and tumor cells. Activated VEGF-VEGFR2 could accumulate Treg cells and control the migration of T lymphocytes [45]. The IL-10R signal on effector T cells and Treg cells is essential to keep immune tolerance [46]. Emerging studies have identified PVR2 as a new immune checkpoint [47].

Of note, this study revealed that LGALS9 and TGFBR1 were upregulated in PC compared to normal tissues. Moreover, we showed LGALS9 and TGFBR1 were significantly associated with the prognosis in PC. Despite the fact that LGALS9 and TGFBR1 were not significantly correlated to the grades, we indeed observed LGALS9 had an upregulated trend and TGFBR1 had a downregulated trend. We thought the limited sample size may contribute to this result. Also, the coexpression plus bioinformatics analysis revealed that immunoinhibitors were involved in regulating multiple inflammatory and immune response-related pathways as previously described. Very interestingly, we found LGALS9 was involved in regulating type I interferon signaling pathway, interferon-gamma-mediated signaling pathway, RIG-I-like receptor signaling pathway, NF-kappa B signaling pathway, cytosolic DNA-sensing pathway, and TNF signaling pathway. We also found that TGFB1 was related to mesoderm formation, cell matrix adhesion, TGF-beta signaling pathway, and Hippo signaling pathway. These pathways had been demonstrated as key regulators of tumorigenesis and immune therapy.

Several limitations should also be noted in this study. First, we showed LGALS9 and TGFB1 had a crucial role in PC with a series of bioinformatics analysis. The further experimental validations of their functions in PC could strengthen our conclusion. Second, more clinical samples should be collected to detect the expression of these immunoinhibitors in PC, which could provide more evidences to confirm their prognostic value.

## 5. Conclusion

Conclusively, our data suggested that immunoinhibitor mRNA level was dramatically upregulated, but negatively correlated with OS for PC. All the data suggested these genes could be used as an emerging prognostic indicator and targets in PC patients. Our findings would give a hint to have a better understanding of the mechanism implicated in PC and stretched out more precise immunotherapeutic treatments for PC prognosis. Nevertheless, more researches and efforts should be contributed to our findings, followed by providing a much more promising clinical strategy for an early diagnosis and prognostic marker in PC therapy.

## Figures and Tables

**Figure 1:** Identification of immunoinhibitor expression pattern in PC. The present study analyzed the expression pattern of 23 immunoinhibitors in PC using TCGA database, including CD160, CD244, KIR2DL1, KIR2DL3, BTLA, CSF1R, HAVCR2, TIGIT, LAG3, PDCD1, VTCN1, PDCD1LG2, LGALS9, CD96, TGFBR1, TGFB1, CTLA4, ADORA2A, PVRL2, IL10, IDO1, IL10RB, and KDR.

**Figure 2:** Increasing expression of immunoinhibitors was observed in PC samples. TGFB1 (a), PVRL2 (b), CSF1R (c), TGFBR1 (d), VTCN1 (e), LGALS9 (f), IL10RB (g), KDR (h), and IDO1 (i) mRNA levels were significantly upregulated in patients with PC compared to normal tissues.

**Figure 3:** Immunoinhibitors were positively correlated to the advanced grade in PC. TISIDB database analysis revealed the expression levels of TGFB1 (a), PVRL2 (b), CSF1R (c), TGFBR1 (d), VTCN1 (e), LGALS9 (f), IL10RB (g), KDR (h), and IDO1 (i) in grade 1, 2, 3, and 4 PC samples.

**Figure 4:** Immunoinhibitors were positively correlated to the advanced stages in PC. TISIDB database analysis revealed the expression levels of TGFB1 (a), PVRL2 (b), CSF1R (c), TGFBR1 (d), VTCN1 (e), LGALS9 (f), IL10RB (g), KDR (h), and IDO1 (i) in stage I, II, III, and IV PC samples.

**Figure 5:** Analysis of the correlation between immunoinhibitor expression and survival time in PC patients. Kaplan-Meier plotter database analysis revealed the correlation between the levels of TGFB1 (a), PVRL2 (b), CSF1R (c), TGFBR1 (d), VTCN1 (e), LGALS9 (f), IL10RB (g), KDR (h), and IDO1 (i) and overall survival time in PC patients.

**Figure 6:** Construction of the coexpression network of immunoinhibitors in PC patients.

**Figure 7:** Assessment of the function of LGALS9 and TGFB1in PC patients. GO (a) analysis and KEGG pathway (b) analysis of LGALS9 in PC patients. GO analysis (c) and KEGG pathway analysis (d) of LGALS9 in PC patients.

## Data Availability

The datasets used during the present study are available from the corresponding author upon reasonable request.
